This article has been retracted.

# Optimization and Simulation of Enterprise Management Resource Scheduling Based on the Radial Basis Function (RBF) Neural Network

**DOI:** 10.1155/2021/6025492

**Published:** 2021-06-29

**Authors:** Ye Wu, Xiaowen Sun

**Affiliations:** School of Business, Macau University of Science and Technology, Macau 999078, China

## Abstract

In the human resource system of modern enterprises, human-post matching big data occupies an important irreplaceable position. With the deepening of the reform of state-owned enterprises, some shortcomings of human-post matching big data have become prominent. The purpose of this article is to solve the current state-owned enterprises. There are a variety of problems with big data in the enterprise, and an effective method is found that can accurately evaluate the degree of human-job matching in state-owned enterprises and provide a scientific basis for the manager of talent and resource allocation to make more rational decisions. Through the radial basis function (RBF) neural network-based big data model of human-post matching evaluation of state-owned enterprises, we scientifically and effectively evaluate the matching degree of the quality and ability of the personnel with the relevant requirements of the position and then help the company to adjust the personnel at any time changes in positions to maximize the efficiency of human resources. In this paper, considering the actual situation of the enterprise, the RBF neural network and the analytic hierarchy process (AHP) method are used comprehensively. Firstly, the AHP is used to obtain the weight of each evaluation index in the human-post matching index system. At the same time, the artificial neural network theory is self-adapting. Learning is helpful to solve the problem that the AHP method is too subjective. The two learn from each other's strong points and combine their weaknesses organically to increase the convenience and effectiveness of evaluation.

## 1. Introduction

Reasonable matching of personnel and positions requires one-to-one correspondence between people's knowledge, experience, and abilities and job requirements. Reasonable matching of human resource big data is the main factor for continuous optimization of human resource management [1]. Talents and positions are the two components of big data matching with people and positions. Among them, talents are the key factor that determines the success or failure of the mixed ownership reform of state-owned enterprises [2]. This article discusses the big data problem of personnel and job matching, which can provide strong theoretical support for the selection of corporate talents. It can not only continuously improve the company's internal human resources big data system but also make the efficiency and accuracy of human resource management in a wide range. Promotion can also provide theoretical guidance for the reasonable allocation of company talents, promote the dual improvement of personal and organizational performance, and promote the healthy and orderly development of the company [3]. Neural network is one of the most widely used classification methods for data mining algorithms. It has solved practical problems in a wide range of fields such as pattern recognition, intelligent robots, predictive evaluation, and economics. It is mainly used in the processing of nonlinear data. It has the functions of associative storage, self-learning, and high-speed search for optimized solutions. The current typical algorithms are RBF neural network and other algorithms [4].

Person-post matching is an important part of human resources big data. Managers are the backbone of state-owned enterprises. The quality of managerial personnel-post matching directly affects the reform process of state-owned enterprises. At this stage, although some state-owned enterprises have also found an irreplaceable position in human resource management and development, in recent years, they have also adopted a variety of methods to attract and retain talents to promote the progress of the company [5]. However, human resource big data not only is an increase in quantity and quality but also requires the ability to rationally use human resource big data. It can effectively allocate personnel and positions, and through reasonable and effective human resource management and development, it can maximize the operational benefits of human resources in the business process in the daily life of the enterprise [6]. Otherwise, once human resources are not well managed and controlled by big data, losses will occur within the state-owned enterprises, resulting in a shortage and waste of state-owned enterprises' human resources. Modern state-owned enterprises mainly adopt traditional algorithms such as the analytic hierarchy process for personnel and job matching, which will cause too strong subjectivity. Therefore, the RBF neural network is added to effectively utilize the powerful self-organization, self-adaptability, and self-adaptability of neural networks. Self-learning ability avoids the disadvantages of too strong subjectivity in the evaluation of traditional state-owned enterprises' personnel-post matching and brings new ideas and methods for state-owned enterprises' personnel-post matching [7].

Based on the research on the big data theory of human resources person-post matching, this paper analyzes the person-post matching branch of the human resource information big data system in detail. Through literature review and summary, it is determined which characteristics of employees are suitable for managers of state-owned enterprises. The evaluation of job status is effective. It objectively analyzes the status quo of management positions in state-owned enterprises, lists out the many factors that can be competent for management positions, and builds an evaluation index system for the matching of basic, middle-, and high-level managers in state-owned enterprises. The job matching evaluation model provides strong theoretical support for the evaluation and selection of human resources. By constructing a scientific and reasonable index system, this article helps state-owned enterprises recognize the real talent needs of management positions, understand the types of qualities that state-owned enterprises need for managers, and help improve the management mechanism of state-owned enterprise management talents. The overall operating efficiency and market competitiveness of the enterprise have been improved.

## 2. Related Work

In terms of human capital investment decision-making, when American economist Tang and Fishwick [8] studied the relevant factors of human capital growth, he once put forward the hypothesis that (1) personal time is only allocated to production and human capital investment; (2) the human capital owned by the individual is only used for production and human capital investment; and (3) the individual already has a certain amount of human capital before the beginning of his career. The rough set is based on classification. Classification is the hierarchical relationship established in the data. These relationships realize the division of data. In terms of the description and processing of uncertainty, rough set theory is more objective for data processing. Based on assumptions, he believed that human capital includes two aspects, flow and stock, and established a human capital growth model using the Cobb–Grass production function. In different research stages, experts and scholars have made their own contributions to the development of marketing theory from different research perspectives. Zhu et al. [9] believed that the essence of marketing management is the “creative adaptation to the dynamic environment” of the enterprise. The task of marketing is to use various means to achieve the best environmental adaptation. Chang and Xu [10] put forward the target market theory on the basis of previous research and believed that “while adapting to the external environment, companies should also develop marketing mix strategies to meet the needs of the target market and achieve the company's goals.” Lv et al. [11] proposed that marketing is the overall system of corporate activities, through pricing, promotion, distribution activities, and various channels to provide products and services to real customers and potential customers. He tried to clarify why and how companies constantly modify their behavior in the market of their choice to enhance adaptability and pointed out that marketing is not just a function; it is a whole process throughout. After entering the 90s, marketing theory has entered a period of great development, with new marketing theories such as relationship marketing, service marketing, network marketing, green marketing, integrated marketing, and knowledge marketing, as well as marketing decision support systems, marketing expert systems, etc. New marketing practices have greatly expanded and enriched marketing management theory. Tang and Cai [12] used years of education to represent general human capital and working years to represent firm-specific human capital. The work conditions of 65 employees of one of Israel's largest municipal companies were evaluated. Empirical studies have found that there is a significant positive correlation between the number of years of education and tenure and the performance of the same group. Groups with higher human capital have higher work performance. Zhao et al. [13] believed that entrepreneurs' transnational experience is a kind of valuable human capital that is difficult to imitate. He collected data on the transnational experience of CEOs of 256 American multinational companies and, on this basis, used empirical methods to prove that the CEO's transnational experience, a special human capital, has a positive and positive effect on corporate performance.

The research content abroad is mainly about how to deal with and get rid of the crisis after a corporate crisis occurs. As for the cause and development process of the crisis, there is a lack of mechanism analysis [14]. The development of macroeconomic early-warning research and the theory of corporate crisis management has promoted corporate early-warning research. Some scholars have studied the early-warning system of small- and medium-sized enterprises and put forward the three most important risk factors of management ability, accounting system, and attitude towards employees [15–18]. Some researchers have made the judgment of a single financial ratio model for the first time, creating a single variable early-warning method. With the establishment of the concept of information flow, some scholars have proposed models that use cash flow information to predict financial distress [19]. It has strong theoretical complementarity with fuzzy mathematics, probability theory, neural network, and other inaccurate problems, and it relies on the theoretical basis that rough sets can deal with incomplete and inaccurate problems. Foreign enterprise early-warning research is based on empirical methods, focusing on corporate functional levels such as financial early warning in content, but there are not many studies on enterprise early-warning principles and the construction of early-warning systems [20]. Domestic early-warning research started relatively late. The main feature of the initial stage of the research is the introduction and specific application of the above methods. The research and application of early-warning management have experienced a process from macroeconomic early warning to enterprise early warning, from qualitative to quantitative [21, 22].

## 3. Construction of the Enterprise Management Resource Scheduling Model Based on the RBF Neural Network

### 3.1. RBF Neural Network Level

Neural network is an operation mode formed by interconnecting nodes or neurons, and each node or neuron is an output function [23–25]. The connection between nodes represents the weight of the signal between two nodes. The output of the model is the way the network is connected. The connection has different weights for different nodes. The network model itself is an approximation of the function. The artificial neural network is also referred to as a neural network or connection model for short. It is an algorithmic mathematical model that simulates the behavioral characteristics of animal neural network and performs distributed and parallel information processing. Different from traditional methods to solve problems, artificial neural networks solve problems through training.  Figure 1 shows the hierarchical relationship of the RBF neural network. The artificial neural network has self-learning and self-adapting capabilities. It can analyze and grasp the underlying laws between the two through a batch of corresponding input-output data provided in advance so that the artificial neural network can learn to be included in the “solution.”

We consider the fully connected multilayer forward network, assuming that *X* and *Y*, respectively, represent the input and output vectors of the network, *Y* represents the actual output of the network and, respectively, represent the number of network input units, hidden units, and output units allowed; then, the input layer, hidden layer, and output layer unit refer to relationship *y*1…*y* − *i*. The output layer and input layer can be expressed as follows:

(1) $$\begin{array}{c} x\left(n\right)=\left\{x_{i}\right\},\;\left(i=1,2,\ldots ,n\right). \end{array}$$

This process continues to circulate, so that the network continuously corrects the connection weight value and finally minimizes the mean square error between the network output result and the expected output vector, so as to find a set of connection weight matrices, and when a new input signal is received, fuzzy calculation and prediction functions are given:

(2) $$\begin{array}{c} u\left(x\right)=\underset{n⟶\infty }{\lim}\sum_{i=1}^{n}a\left(i,j\right)\cdot x\left(i\right)-b,\;i=1,2,\ldots ,k, \end{array}$$

(3) $$\begin{array}{c} v\left(x\right)=\underset{n⟶\infty }{\lim}\sum_{i=1}^{n}a\left(j,i\right)\cdot x\left(i\right)+b,\;i=1,2,\ldots ,k. \end{array}$$

According to the existing research results, the transfer function between the input layer and hidden layer neurons in the RBF neural network model can usually be a sigmoid function, which is also called a squashing function or a logistic function. Its general expression is as follows:

(4) $$\begin{array}{c} \frac{\text{d}u\left(x\right)}{\text{d}x}+\frac{\text{d}v\left(x\right)}{\text{d}x}=y\left(x\right)\cdot x\left(i\right). \end{array}$$

In the formula, *R* is the number of neurons in the input layer, *X* is the row vector composed of the values of the neurons in the input layer, and *W* is the position of each neuron in the hidden layer in the input layer. A column vector is composed of corresponding weight values on each neuron. Through the calculation of the above formula, the neurons in the hidden layer can output a value in the range of [0, l] and then further transfer to the output layer neuron. The transfer function of the RBF neural network model between the hidden layer and the output layer neurons is usually a linear function, and its general expression is as follows:

(5) $$\begin{array}{c} \frac{w\left(i,j\right)-w\left(i,j-1\right)}{x\left(i,j\right)+w\left(i,j-1\right)}=\int f\left(x\right)x\text{d}x, \end{array}$$

(6) $$\begin{array}{c} \left\{\begin{array}{cc} \alpha \cdot w\left(i\right)+\beta =1, & i>j,\\ \alpha \cdot w\left(j\right)-\beta =0, & i<j. \end{array}\right) \end{array}$$

Among them, *k* is the magnification factor (slope) and *b* is the displacement (intercept). It is easy to know that the domain and value range of this function are both the set of real numbers R. Through this function, the output layer neuron can linearly transform the value of the hidden layer neuron and then cooperate with the established teacher signal and calculate its mean square error.

### 3.2. Resource Scheduling Algorithm

The feedforward network composed of nonlinear transformation units can simulate the human brain's learning process, thinking mode, and neural signal conduction mode, through the early input of teacher signal for “training”; the signal is passed through the input layer from the input variable of the input layer of the network:

(7) $$\begin{array}{c} g\left(x\right)=\left\{\begin{array}{cc} \exp\left(x\right)-\exp\left(-x\right), & x>0,\\ \exp\left(x\right)-\exp\left(-x\right), & x<0, \end{array}\right) \end{array}$$

(8) $$\begin{array}{c} h\left(i,j\right)=\left[\begin{array}{ccc} w\left(1,1\right) & 0 & 0\\ 0 & \ldots & 0\\ 0 & 0 & w\left(i,j\right) \end{array}\right],\;\left(i,j=1,2,\ldots ,k\right). \end{array}$$

After processing, it is transferred to the hidden layer, and the neurons in the hidden layer pass through the transfer function (also called the activation function) one by one.  Figure 2 shows the resource scheduling algorithm. After the calculation, the result is processed and passed to the output layer through the connection weight *M* between the hidden layer and the output layer and then compared with the expected output signal (vector) given in advance, such as finding the network output result and the expected output. If there is a large error between the vectors, the network feeds back the error, uses a certain method to change the aforementioned connection weight W, and then adjusts the network output result according to the new weight value and compares it with the expected output vector.

As the scale or complexity of the problem increases, the design of the ANN may become more complex. Many people who are interested in applying ANN are often intimidated by it. Evolutionary computing, with its inherent advantages-group optimization search, provides a new way for the design of ANN. Preliminary research has shown unique advantages. The pruning method is to learn from an initial network with a structure larger than the smallest solution network. In the network training process, the obtained satisfactory network is gradually deleted according to certain performance criteria, and unnecessary connections or nodes are deleted. When the performance of the network deteriorates, the training is stopped, and a satisfactory learning network is obtained. The learning network structure obtained by the pruning method is streamlined and has good performance. The problem is that, first, it is difficult to select the size of the initial network. To get a suitable initial network, it is necessary to use trial and error methods. In addition, the same problem as the construction method is that the obtained learning network is likely to be a local optimal solution.

### 3.3. Network Model Weight Update

The evolutionary learning of connection rights has many advantages. For example, evolutionary learning does not depend on derivative information, has a high degree of parallelism, and is good at dealing with global optimization problems where the solution space is complex and multipeak terrain. The RBF algorithm specifies the number of categories as *k* and clusters the sample set. The clustering result is expressed by clustering centers. Based on the given clustering index function (or the criterion of clustering effect), the algorithm adopts iteration. In the updated method, each iteration process is carried out in the direction of decreasing the value of the index function, and the final clustering result makes the value of the index function a minimum value and achieves a better clustering effect. However, there is a permutation problem in evolution; that is, a network structure in the solution space may correspond to multiple individuals in the coding space. The difference between these individuals is only that the coding representation is different, which leads to the failure of exchange operations.  Figure 3 shows the weight ladder diagram of the network model under the RBF neural network.

The analytic hierarchy process divides many index factors into the highest level, the middle level, and the lowest level. The highest level is also called the target level, which represents the final goal of the evaluation; here is the overall marketing risk. The middle level represents the intermediate level indicators involved in reaching the final goal of the evaluation, also called the criterion level, which can be composed of several levels. This refers to five aspects: competition risk, collaboration risk, public risk, product risk, and marketing organization management risk; the key is the bottom-level specific evaluation index, that is, the establishment of subfactor indicators. This level is also called the program level.

The learning algorithm of the evolutionary neural network is constantly evolving.  Figure 4 shows the framework of the enterprise management resource scheduling model based on the RBF neural network. The traditional RBF algorithm has a strong dependence on the initial center selection, and the value needs to be determined in advance. According to the characteristics of the lead time estimation problem, the use of an improved algorithm based on a fuzzy similarity matrix can alleviate the initial value dependence of the traditional algorithm, automatically determine the number and center of clusters, and also greatly reduce the efficiency and effect of the algorithm. Moreover, many people integrate heuristic knowledge or information into the learning algorithm of the evolutionary neural network, which improves the efficiency of evolutionary learning. The evolution part of neural network structure includes selection of structural variant individuals, structure (hidden unit, connection) addition, deletion and mutation, individual network parameter initialization: individual connection weight learning, structure evaluation mechanism. After structural mutation, it is possible to judge structural learning only after the evolutionary learning of connection weights. Therefore, in the process of evolving neural networks, connection weight evolution learning is the “inner loop” of the structure evolution learning process, and it is indispensable. Based on the above analysis, it can be considered that the RBF neural network model established in this article has basically reached the expected error level after 108 cycles of training and can be used for simulation and prediction. In the process of neural network evolutionary learning, the evolutionary learning rules or the control parameters in the algorithm are not static. The evolution of learning rules can be carried out with the support of an expert system, or it can be completed through machine self-learning and self-adaptation.

## 4. Application and Analysis of the Enterprise Management Resource Scheduling Model Based on the RBF Neural Network

### 4.1. RBF Neural Network Parameter Optimization

In the RBF artificial neural network learning, the sigmoid function is used as the output. Due to the limitation of computer operations, the evaluation expectation value only takes the range of (0.5, 1), and the final evaluation result is within the range of (0.5, 1). We carry out 5 equal divisions, which does not affect the evaluation results. In the enterprise ecological evaluation, first evaluate the evaluation objective, including the stability of the enterprise's internal environment; the enterprise's environmental adaptability, the status of the enterprise, competitiveness, and enterprise innovation and development capability are evaluated. Then, these four subobjectives are used as the evaluation elements of the evaluation objective to evaluate the enterprise ecology. Since there are five largest eigenvalues in the correlation coefficient matrix, which are 8.733, 5.875, 4.432, 2.668, and 2.199 (this article sets the number of common factors to be extracted in the factor extraction dialog box to 5), the extracted five common factor features are all greater than 2. Because, in the data used in this article, the dependent variable (InvestDem) is divided into 4 levels, this article uses the Multinomial Logistic Regression in SPSS 15 to test and set the dependent variable to InvestDem and set the covariates to the remaining 7 indicators (all discrete categorical variables).  Figure 5 shows the line chart of the correlation coefficients of enterprise evaluation elements.

For factor 1, the indicators on which the load value is greater than 0.8 are as follows: return on net assets growth rate, earnings per share growth rate, sales profit rate growth rate, return on net assets, net sales profit rate, return on total assets. For factor 2, the indicators on which the load value is greater than 0.8 are as follows: shareholder equity growth rate, net asset growth rate, net asset growth rate per share, and total assets growth rate. For factor 3, the indicators on which the load value is greater than 0.8 are as follows: current ratio, quick ratio, and asset-liability ratio. For factor 4, the indicators on which the load value is greater than 0.8 are as follows: accounts payable ratio, sales real growth rate, and accounts receivable turnover rate. For factor 5, the indicators on which the load value is greater than 0.8 are as follows: sales profit rate and sales revenue growth rate.  Figure 6 shows the histogram of the amount of human resources information. The layer numbers 1–4, respectively, represent the input layer, data layer, analysis layer, and output layer. This paper divides the enterprise ecological evaluation into five evaluation indicators, which are the stability of the enterprise's internal environment, the adaptability of the enterprise to the environment, the status quo of the enterprise, the core competitiveness of the enterprise, and the ability of innovation and development of the enterprise. Each subindicator is divided into several two secondary indicators. In order to make the RBF artificial neural network enterprise ecological evaluation results comparable, the selected enterprises are enterprises in the same industry.

At this time, you can keep those indexes that are greater than a certain critical value in a principal component combination coefficient and delete other indexes. After finite principal component analysis, all remaining indexes can reach the retention standard. These retained indicators constitute an indicator system. In practical applications, the critical value of the load factor and the number of principal component analyses can be flexibly adjusted according to the value of the factor load matrix and the expected number of principal components. Generally, the load value of the main index is required to be no less than 0.5. In the experiment, the data in the column of “output value after sorting” is merged from “Node l output value” and “Node 2 output value” after rounding, and the “expected value” data is the two columns of “Node l” and “Node 2” of samples numbered 4-5. According to the rules listed in the paper, they are converted into “network prediction results” and “expected results” and compared. In this paper, the parameter 0.8 is selected as the critical value of the load coefficient for dividing the primary and secondary indicators, and finally, a new early-warning evaluation indicator system composed of 18 indicators is obtained.

### 4.2. Enterprise Management Resource Data Simulation

This paper uses the neural network toolbox of MATLAB engineering calculation software to design, train, and test the established early-warning model of the RBF neural network. In this paper, the number of hidden units is set to 3. The number of output units is 1, and the learning step length is 0.1. Input the data into the learning program of the REF artificial neural network, and it will reach the set output error after 33618 times. We input each evaluation index of the evaluation sample, respectively, to obtain the enterprise ecological evaluation result of the enterprise. In the learning process, since the evaluation result has a certain error with the expert's expected value, fuzzy processing is adopted for the evaluation result. Let the evaluation result value be *Y*. (1) *Y* ≤ 0.50 is the first level: (2) 0.50 < *Y* ≤ 0.6 is the second level; (3) 0.60 < *Y* ≤ 0.70 is the third level: (4) 0.70 < *Y* ≤ 0.80 is the fourth level; and (5) *Y* > 0.80 is grade five.

In this study, 31 indicators (X1 to X31) of 26 companies were used as the research sample data. After direct entry and indirect calculation, the specific values of 31 indicators are obtained.  Figure 7 shows the scoring curve of early-warning indicators for different sample points. Among them, the top ten (0–10) companies are electronic companies, and their related index data will be used as the training data set of the model; the eleventh to fourteenth (11–14) related indexes of the four companies. The data will be used as the detection data set of the model, and the relevant index data of the following twelve (15–26) companies will be used as an example of early-warning model analysis. Using statistical analysis software SPSS 12.0, the original data of the above indicators of 26 companies were tested. The simulation shows the changing trend of the value during the training process. Since the RBF neural network uses an algorithm, the value in the figure is an adjustment parameter in the LM algorithm, which is used to adjust the weight in two adjacent iterative calculations. The change of this parameter after about the 45^th^ training is small, indicating that the connection weight within the network has a small change, indicating that the network has entered a more stable state. The results of the KMO sampling adequacy test and the Barnett method sphericity test are shown in the paper. The KMO sampling adequacy test value is greater than 0.5; it can pass the Bartnet method of sphericity test (significance level 0.001). The two test results show that the data can be used for principal component analysis.

### 4.3. Example Application and Analysis

In order to fully reflect the development trend of high-tech, the proportion of R&D expenditure in sales revenue and the proportion of scientists and engineers in the total number of employees can be selected from two aspects: technology intensity and economic benefit level, per capita profit and tax rate, and total labor productivity and other indicators, using neural network models to comprehensively evaluate the technology intensity and economic efficiency of high-tech enterprises. At the same time, the correlation coefficient matrix of 31 indicators is calculated. Through the correlation coefficient matrix table, it can be found that the correlation between some indicators is very large (the absolute value of the correlation coefficient is greater than 0.8), and the correlation between some indicators is very small (the absolute value of the correlation coefficient is less than 0.5); further processing of high marketing early-warning indicators directly enters the marketing early-warning system, which will inevitably cause information redundancy. Because there is indeed a greater degree of correlation between some primary indicators, it can be judged that it is necessary to integrate the indicators to solve the problem of information overlap between early-warning indicators.  Figure 8 shows the dependence of resource scheduling score on the number of neural network training.

When evaluating an enterprise using a neural network model, first take the maximum and minimum values of all indicators in all the evaluated enterprise objects as the two learning samples and take the national high-tech enterprise identification sample as the third learning sample. The expected outputs corresponding to these three learning samples are 1, 0, and 0.6, respectively. Using these three sets of data as learning samples for learning, the final weights and thresholds can be obtained. Finally, the obtained weights and thresholds can be used to evaluate the enterprises that need to be evaluated. When using the neural network model for evaluation, the original data is normalized using the aforementioned method.

According to the statistical significance of the degree of commonality of variables, it plans the contribution of all common factors to the total variance, and it shows the percentage of information that all common factors reflect the original variable.  Figure 9 shows a box plot of variance statistics for the number of neural network indicator layers. For example, after extracting the common factor, the commonness of the variable X3 is 0.971; that is, the extracted common factor makes a 93.1% contribution to the variance of the variable X3. From the values obtained after extracting the common factors, it can be seen that the commonality of each variable is relatively large, indicating that when the variable space is transformed into the factor space, more information is retained. It is found through comparison that, among the 10 samples used for simulation testing, only the network output results of sample 4 and sample 5 are not consistent with the expected results, and the network accuracy rate reaches 80%, which proves that the network design is reasonable and the network prediction result is basically credible; it can be used for the company's analysis and judgment of employees' cross-cultural training needs. Therefore, the effect of using principal component analysis to extract common factors is significant. The number of layers of the model is three layers, namely, the input layer, the hidden layer, and the output layer. The input node is set to four according to the number of indicators, and the output layer is one node. The number of hidden layer nodes is set to 7 according to trial calculations. The value of the two learning parameters is 0.5, and the learning accuracy is 0.0001.

Figure 10 shows the linear fit of the neural network model data output value. The evaluation results show that there are 10 companies with a comprehensive evaluation score of 0.6 or more. The results of the national standard evaluation are basically the same. An electronic information company and a technology company failed to meet the standard because the national standard evaluation is a single-target screening and did not give a proper comprehensive reflection of all evaluation indicators; the number of scientists and engineers of these two companies accounted for the proportion of the total number of employees and the labor productivity of all employees. The neural network model objectively reflects the actual situation of these two indicators. Combining these two indicators with other indicators for a comprehensive evaluation, the evaluation results are more reasonable.

## 5. Conclusion

This paper takes the state-owned enterprise company as an example to carry out a case analysis and obtains the accuracy and operability of the human-post matching evaluation model, which can provide a theoretical support plan for the staffing of state-owned enterprises. The RBF neural network in data mining is used to study regional personnel input, economic output, and energy consumption. This article separately studies the three main influences of the development zone. And the test results have been analyzed and studied, to provide technical support for the division of the green development of enterprises in the development zone. It has certain advantages in solving such problems and can maximize the role of human resources, expand the construction of the talent team for corporate management positions, and also play a guiding role in the six major modules of corporate human resources. The experimental results prove that the accuracy is 86.3%, 80.90%, and 86.36%, respectively. The RBF neural network algorithm can initially divide the enterprises in the development zone, using the complementarity of the rough set and the RBF neural network to extract and determine the data attribute weight factors and determine the basic development zone enterprises through the comprehensive measurement of the weight of each attribute. The comprehensive weight of the development management data is 0.55, 0.25, and 0.2, and the weight is combined with the RBF neural network algorithm to apply it to avoid the RBF neural network from being prone to minimize the phenomenon in the calculation process. Secondly, according to the characteristics of the company and the specificity of listed companies and the actual situation of the data and information obtained, some adjustments were made to the constructed marketing early-warning indicators. The statistical analysis software SPSS 12.0 was used to compare the above indicators of 26 companies. The original data was tested and the principal component analysis method was introduced, and 18 indicators were finally confirmed as the early-warning indicator system for this thesis research. We carried out the application of the rough set RBF neural network algorithm in the classification of the green development of enterprises. The key to the rough set RBF neural network is the structural information of the data. The structural information in the whole derivation process is the attribute weight. This article applies the attribute weight to the RBF neural algorithm, but the determination of the weight itself depends on the inherent nature of the data. In the follow-up research, try to introduce other algorithms. The rough set RBF neural network algorithm can efficiently and accurately realize the prediction and analysis of the green development of enterprises in the development zone. It shows that the RBF neural network algorithm is useful for development and the division of district enterprises is feasible.

## Figures and Tables

**Figure 1:** Hierarchical relationship of the RBF neural network.

**Figure 2:** Resource scheduling algorithm.

**Figure 3:** Network model weight ladder diagram under the RBF neural network.

**Figure 4:** The framework of the enterprise management resource scheduling model based on the RBF neural network.

**Figure 5:** Line chart of correlation coefficients of enterprise evaluation elements.

**Figure 6:** Histogram of the amount of human resources' information.

**Figure 7:** Scoring curve of early-warning indicators for different sample points.

**Figure 8:** The dependency of the resource scheduling score with the number of neural network training.

**Figure 9:** Box plot of variance statistics of the number of neural network index layers.

**Figure 10:** The linear fitting of the output value of the neural network model data.

## Data Availability

The data used to support the findings of this study are available from the corresponding author upon request.
